The article "Short Sequence Chinese-English Machine Translation Based on Generative Adversarial Networks of Emotion" was published in 2022. Journal: Comput Intell Neurosci.

# Short Sequence Chinese-English Machine Translation Based on Generative Adversarial Networks of Emotion

**DOI:** 10.1155/2022/3385477

**Published:** 2022-05-31

**Authors:** Hua Wang

**Affiliations:** School of Journalism, Nanjing University of Finance & Economics, Jiangsu, Nanjing 210000, China

## Abstract

With the steady growth of the global economy, the communication between countries in the world has become increasingly close. Due to its translation efficiency and other problems, the traditional manual translation has gradually failed to meet the current people's translation requirements. With the rapid development of machine-learning and deep-learning related technologies, artificial intelligence-related technologies have affected various industries, including the field of machine translation. Compared with traditional methods, neural network-based machine translation has high efficiency, so this field has attracted many scholars' intensive research. How to improve the accuracy of neural machine translation through deep learning technology is the core problem that researchers study. In this paper, the neural machine translation model based on generative adversarial network is studied to make the translation result of neural network more accurate and three-dimensional. The model uses adversarial thinking to consider the sequence of emotion direction so that the translation results are more humanized. We set up several experiments to verify the efficiency of the model, and the experimental results prove that the proposed model is suitable for Chinese-English machine translation.

## 1. Introduction

Since the twenty-first century, the economic level of all countries in the world has been greatly improved. In the context of economic globalization, cross-language communication between people of all countries has become more and more frequent. Different nations have their own customs and cultures, and there are great differences in language expression. How to communicate effectively across languages is a problem that must be faced and solved. Due to its translation efficiency and other problems, the traditional manual translation has gradually failed to meet the current people's translation requirements. Therefore, many people turn their attention to Machine Translation, which is an important branch of natural language processing. Machine translation is to generate the target language with the semantics of the source language unchanged through relevant computer and algorithm and other techniques. That is, to achieve equal conversion from one natural language to another [1, 2].

In the initial stage of machine translation research, the implementation of translation is mainly through the use of rule-based methods. Linguists manually compile translation rules between source language and target language, that is, rules that enable conversion between two natural languages, and then input these formulated translation rules into the system [3]. Although the method that generate conversion rules between source and destination languages has made great progress, this method almost completely depends on the quality of language rules established by linguists, and it has certain limitations in practical application. Moreover, due to the problems such as its too extensive coverage and the direct relationship between language and national culture, it is difficult to list the translation rules between source language and target language. Therefore, the failure to obtain a complete set of language rules [4, 5] is the main problem faced by rule-based machine translation. IBM put forward the Statistical Machine Translation model in 1993. Statistical Machine Translation mainly adopts the way of word alignment between source language and target language. Statistical Machine Translation mainly obtains the conversion rules between two natural languages by learning the corpus, without the need to make conversion rules manually. However, there are still many problems in Statistical Machine Translation [6]. It relies too much on the learning of the model in the corpus and has high requirements on the accuracy of the processing steps such as word alignment, word segmentation, and translation rule extraction [7].

The article "Short Sequence Chinese-English Machine Translation Based on Generative Adversarial Networks of Emotion" was published in 2022. Journal: Comput Intell Neurosci.

In recent years, with the continuous maturity of artificial intelligence technology and the rapid development of machine learning and deep learning-related technologies, deep learning has gradually been combined with different fields. How to improve the accuracy of neural machine translation through related deep learning technology is also a problem that researchers have been studying [8, 9]. Deep learning techniques are used to deal with natural language problems so that some problems faced in natural language processing have been well solved and good results have been achieved. The application of deep learning technology provides many ideas and methods for improving the accuracy and efficiency of machine translation. At present, deep learning technology is mainly used in two models in the machine translation [10]. The first is the Statistical Machine Translation model framework, which adopts neural network to improve and optimize the language model, sequencing model, and other key modules in the model framework. The second method is to construct the encoder and decoder through neural network, and use the end-to-end neural network machine translation model to realize the translation and conversion from source language to target language [11, 12]. With the deepening of research, more and more neural network machine translation algorithms are proposed.

The article "Short Sequence Chinese-English Machine Translation Based on Generative Adversarial Networks of Emotion" was published in 2022. Journal: Comput Intell Neurosci.

## 2. Related Work

### 2.1. Rule-Based Machine Translation

With the birth of computers in the middle of the last century, machine translation began its exploration [13]. In 1954, IBM used the computer to translate several simple Russian sentences into English for the first time. Its translation system consists of six translation rules and 250 words [14, 15]. This experiment shows that the process of machine translation can be realized by using the method based on dictionaries and translation rules. Although it was only a preliminary success, it aroused the enthusiasm of machine translation research in the Soviet Union and other European research institutions. It greatly promoted the research progress of early machine translation. However, machine translation was completely rejected in 1966 by a report titled LANGUAGE AND MACHINES, and machine translation research suffered a setback at that point [16, 17]. With the increasingly close exchanges between countries, the communication barriers between different languages become more and more serious, and people's demand for machine translation is more and more intense. At the same time, the development of corpus linguistics and computer science has provided new possibilities for machine translation. Since then, Machine Translation has entered a period of rapid development. After decades of evolution, it has formed three stages from Rule-based Machine Translation to Statistic Machine Translation and then to Neural Machine Translation [18–20].

The earliest machine translation method is rule-based machine translation, which realizes the conversion between source language and target language by making relevant translation rules. The process of rule-based machine translation mainly includes three steps: source language parsing, language conversion, and target language generation [21]. The first step is to parse the input source language to obtain the structural representation of the source language. The second step is language conversion. Transform the structural representation of the source language into the structural representation of the target language through the formulated translation rules. In the third step, the representation of the target language is generated into the target language by processing the corresponding rules. Early rule-based machine translation methods require manual transformation rules. Although they have high-translation accuracy for a small number of sentences, their coverage is limited, the system robustness is poor, and is very sensitive to noise in rules. The rule-based machine translation method can perform machine translation to a certain extent, but its application is very limited. This translation method almost completely depends on the language rules established by linguists, which has certain limitations in practical application. Moreover, due to the extensive and profound language, it is difficult to list all the rules contained in various kinds of language. Therefore, the inability to obtain a complete set of language rules is the main problem facing rule-based machine translation research.

The article "Short Sequence Chinese-English Machine Translation Based on Generative Adversarial Networks of Emotion" was published in 2022. Journal: Comput Intell Neurosci.

### 2.2. Machine Translation Based on Statistics

In order to solve the problems of rule-based machine translation, statistical machine translation has become the representative method of machine translation research. A landmark event was the launch of Google's free online automatic translation system, also known as Google Translate [22], which really brought the “high-flying” technology of machine translation into people's lives. Statistical machine translation is a data-driven approach that designs probabilistic models on large-scale parallel corpora to achieve automatic translation from source language to target language. Early statistical machine translation was word-based, learning model parameters from words in the corpus. Later, phrases were used as the basis to learn model parameters, and now syntax is used as the basis to build syntactically based statistical machine translation model to further improve translation accuracy. Statistical machine translation model is one of the most widely used machine translation models. This is because statistical machine translation models have excellent translation results in machine translation in unbounded domains.

Statistical machine translation model is to obtain the parameters required by the relevant translation model through the statistical analysis and learning of a large number of parallel corpus, and then to construct the statistical translation model, and then to use the model for translation. Koehn et al. took words as the basic unit of statistical machine translation model, extracted corresponding words of original language and target language from corpus, and proposed phrase-based statistical machine translation model [23]. Och and Ney proposed statistical machine translation based on the maximum entropy model and constructed the machine translation model through the log-linear model [24]. Later, the processing unit of the translation model is extended to include words, and a phrase-based statistical machine translation model is proposed [25]. All of the above statistical machine translation methods are syntactically based and take syntactic structure as the basic translation unit to construct translation models. Although the basic organizational structure of a sentence can be displayed through the syntax tree, the specific semantic information of the sentence cannot be expressed, which makes it difficult for the final translation to correctly represent the original sentence semantics. People gradually turn their attention to the semantic understanding of source language and target language in machine translation. In order to increase the differentiation of translation rules, Aziz et al. integrated the semantic information generated by the source language as a feature into the existing translation model, and marked the nonterminal symbols in the syntactic translation model to a certain extent through the semantic role information [26]. Wu and Fung preprocessed the translation process to realize the utilization of semantic information, reordered the candidate translation list, and marked semantic information with semantic roles [27]. Zhai et al. [28] through the predicate meta-structure made the statistical machine translation model maintain the semantic information of the original text to the maximum extent, made the semantics of source language and target language more similar, and established a semantic translation model based on the transformation of predicate meta-structure.

The article "Short Sequence Chinese-English Machine Translation Based on Generative Adversarial Networks of Emotion" was published in 2022. Journal: Comput Intell Neurosci.

The charm of language lies in the fact that different words have different meanings in different situations. However, in the process of translation, these traditional machine translation models ignore the influence of contextual information on sentence semantics, ignore the context in which the sentence exists, and only focus on the translation of the sentence, which results in the lack of structural rationality and semantic coherence. Therefore, many researchers conduct machine translation research based on the whole article as a translation unit. Xiong et al. [29] proposed a statistical machine translation model based on topic transformation in order to improve the quality of discourse-level statistical machine translation. Gong et al. maintained semantic consistency of the same words and phrases in the whole document through semantic caching technology based on cohesive properties [30]. Tu et al. made a preliminary exploration of the discourse translation framework model based on discourse and proposed a statistical machine translation model that takes the rhetorical structure of discourse as the basic translation unit [31]. Statistical machine translation also has some problems. The independent parameter model structure makes the parameters of the translation model independent, which leads to the situation that the translation model cannot consider the relevance between words, leading to the existence of sparse problem. The process of parameter optimization and training of translation model is independent and not unified. Since learning is carried out in a corpus, statistical machine translation is dependent on the corpus, and the quality of the corpus will directly affect the final translation result. Without in-depth analysis of the source language, if the model does not deal with syntactic and semantic components, it ignores the connection between words and context, which results in the inability to deal with long-distance dependence, resulting in semantic incoherence and unreasonable semantics [32].

The article "Short Sequence Chinese-English Machine Translation Based on Generative Adversarial Networks of Emotion" was published in 2022. Journal: Comput Intell Neurosci.

### 2.3. Neural Network Machine Translation

With the development of deep learning theory, researchers have found that deep learning-related technologies can better solve these problems in statistical machine translation. Neural machine translation technology originated from the neural network probabilistic language model proposed by Bengio et al. in 2003 [33]. It represents discrete characters into continuous dense distributed vectors through neural networks, which effectively alleviates the problem of data sparsity. In 2013, Kalchbrenner and Blunsom et al. [34] from Oxford University constructed an encoder–decoder structure by using CNN and RNN. As an encoder, convolutional neural network (CNN) can obtain historical information and process variable length strings. As a decoder, recurrent neural network (RNN) can directly model translation probability. In earlier studies, deep neural network was only used as an auxiliary method for language modeling, while their study was completely composed of deep neural network, which marked the independent application of deep learning methods in machine translation. Subsequently, Sutskever et al. in Google team proposed RNN-RNN model on the basis of the former, which became the general Sequence-to-Sequence model later. The model uses recurrent neural network as the backbone network of an encoder and a decoder. Cho et al. [35] proposed that Gated Recurrent Unit (GRU) could replace LSTM to handle machine translation tasks. GRU is actually an optimization of LSTM, which simplifies the internal structure, reduces training parameters, and improves training efficiency. Sequence-to-sequence structure, understood abstractly, generates a semantic space. Source language and target language are mapped to this semantic space through neural network training. The more semantically similar words are, the closer they are in the semantic space. In 2014, Bahdanau of Youngor University in Germany proposed attention mechanism, which effectively solved this problem and brought machine translation to a new height [36]. They gave the “S-S” model ability to distinguish, so that it pays attention to the more relevant input information. The attention mechanism is essentially a small neural network trained at the same time as the S-S network. Luong et al. from Stanford proposed many variations of attention mechanism, which further enhanced the representational ability of attention mechanism. After the attention mechanism is introduced, the long-distance dependency problem can be better dealt with. The influence of the previous word on the current word can be obtained through the attention weight, and the representation vector of the current word can be better generated.

The article "Short Sequence Chinese-English Machine Translation Based on Generative Adversarial Networks of Emotion" was published in 2022. Journal: Comput Intell Neurosci.

With the proposal of attention mechanism [37] and the rapid development in the field of image, attention mechanism is gradually combined with natural language processing. Especially in machine translation, attention mechanism is introduced between the current state of the target language sequence and the hidden layer state of the source language sequence. The matching degree of these two states is measured by attention weight, so as to obtain a better representation vector of the target language. The problems of long-distance dependence and incomplete representation of vector information are effectively solved [38]. Mi et al. used punishment to improve the translation effect. If the completed part of the translation received too much attention, it would be punished and reward the unfinished part of the translation [39]. In order to obtain better translation results, Tang et al. selected the required rules through the attention mechanism in the translation process, but it also caused high-time complexity [40]. Researchers have never stopped improving the neural machine translation model and have made some achievements in improving the memory capacity of the model and expanding the depth of the translation model [41].

Although neural machine translation has surpassed statistical machine translation in many publicly evaluated translation tasks, its actual translation quality is far from the level of human expert translation, and the model of neural machine translation still needs to be optimized. Compared with phrase-based or rule-based statistical machine translation, neural machine translation lacks the basis of theoretical explanation, because deep learning itself is a “black box” approach. Besides, the complex network structure and the large number of parameters mean the need for large-scale and high-quality parallel corpus pairs. However, high-quality parallel corpus pairs are often missing among many less-popular languages. From the cyclic neural network based on attention mechanism to the convolutional neural network based on attention mechanism to the current mainstream Transformer model based on self-attention mechanism, Transformer's parallel input combined with the self-attention mechanism makes the actual distance between the input words as 1. It effectively alleviates the long-distance dependence problem. At the same time, the computing speed is greatly improved. However, this also leads to inferior representational ability of local information as RNN and CNN, and damages relative location information. In addition to the Transformer model, there is still a lot of room for improvement in the neural machine translation model.

The article "Short Sequence Chinese-English Machine Translation Based on Generative Adversarial Networks of Emotion" was published in 2022. Journal: Comput Intell Neurosci.

## 3. Network Framework

Bi-LSTM and Transformer are widely used in various fields of artificial intelligence. How to further improve the translation effect of Bi-LSTM and Transformer neural machine translation models which introduce attention mechanism that is the focus of this paper and also the innovation of this paper. In this paper, the generative adversarial network is added to the neural machine translation model. The generator adopts Bi-LSTM and Transformer neural machine translation models, respectively. The discriminator uses convolutional neural network to discriminate the translation results and generates feedback to act on the generator. Through the idea of generating antagonism, the effect of generator is improved, that is, the final translation effect of the machine translation model is improved. Language is an important means of expressing emotions. Confrontational training methods can judge positive or negative emotions, and such translation results have emotional effect also.

Based on the end-to-end neural machine translation model, the neural machine translation model adopts the encoder-decoder framework structure. Encoder-decoder model framework is used to encode and decode variable sequences of input and output. In the frame of the model of the encoder and decoder, the decoder corresponds to the output sequence, and the encoder corresponds to the input sequence. The decoding stage decodes the whole target language sequence by maximizing the probability of prediction sequence, and the coding stage encodes the whole source language sequence into a vector. The encoder-decoder framework mainly realizes the probability prediction of target language through the encoding and decoding process of encoder and decoder. Assuming that the source language sequence is *X* ∈ [*x*_1_, *x*_2_, ...*x*_*n*_] and the target language sequence is *Y* ∈ [*y*_1_, *y*_2_, ...*y*_*m*_], the probability calculation of generating the target language is shown in formula (1). The generation probability of each target language vocabulary is calculated by softmax function as shown in formula (2).

(1) $$\begin{array}{c} P=\left(y_{1},y_{2},...,y_{m}|x_{1},x_{2},..,x_{n}\right)=\prod {}_{t=1}^{t=m}p\left(y_{t}|c,y_{1},...,y_{t-1}\right), \end{array}$$

(2) $$\begin{array}{c} p\left(y_{t}|x,y<t;\theta \right)=\frac{\exp\left(\phi \left(y_{t},x,y<t,\theta \right)\right)}{\sum_{y\in Y}\exp\left(\phi \left(y,x,y<t,\theta \right)\right)} \end{array}$$

where *C* is the vector used to represent the source language sequence, contains the relevant information of the source language sequence, and is the vector with fixed dimensions generated by the encoder stage. The *ϕ* function defines the possibility of generating the current target language term *y*_*n*_ from the source language as well as the generated target translation. The purpose of introducing the softmax function is to generate the probability distribution of the target word and to ensure that the function value satisfies the probability distribution. *c*_*s*_ represents the source language context vector representation, *c*_*t*_ represents the target language context vector representation, *Y* represents the target language, and *v*_*y*_ represents the word vector representation of the target language. The known source language sentences and generated target language sentences are used to predict the current probability of the target word. Since the source language sentences and generated target language sentences are very sparse, neural machine translation uses continuous representation to model the conditional probability of the current word in the target language.

The article "Short Sequence Chinese-English Machine Translation Based on Generative Adversarial Networks of Emotion" was published in 2022. Journal: Comput Intell Neurosci.

### 3.1. RNN Neural Translation Model

Owing to the network structure of Recurrent Neural Networks, which perfectly fits the sequence problem, it can process the input sequence of any length in theory. In the process of processing the sequence problem, Recurrent Neural Networks can store the time sequence information and store the historical information of the time sequence through the implicit state. Therefore, the structure of cyclic neural network is generally adopted to deal with sequence problems. The output of the recurrent neural network is a hidden layer state, which is used when the current layer processes the next layer, and each layer outputs to the next layer. This structure enables the recurrent neural network to process the input sequence data well, and to process the data samples with contextual dependencies. The hidden layer state at each moment is a functional representation of all the hidden layer states at the previous moment. According to the time sequence, the schematic diagram of the cyclic neural network is shown in Figure 1.

As shown in Figure 1, the input in the network at time *t* consists of the hidden layer state *h*_*t*−1_ at the previous moment and the input *x*_*t*_ at the current moment. The hidden layer state *h*_*t*_ at the current moment can be calculated by *h*_*t*−1_ and *x*_*t*_. The hidden layer state *h*_*t*_ is computed repeatedly until all inputs are complete. In general, the zero vector is used to represent the initial state of the hidden layer. If the neural network contains only one hidden layer, the activation function of the hidden layer will generally adopt sigmoid function, which is represented by *σ*. For a batch data with *n* samples, assuming that the length of the hidden layer is *h* and the dimension of the feature vector of the sample data is *X*, the output representation of the hidden layer is shown in formula (3):

(3) $$\begin{array}{c} H=\sigma \left(XW_{xh}^{T}+b_{h}\right),X\in \left(R^{n\times x}\right), \end{array}$$

where *b*_*h*_, *w* represents the bias vector parameters and weights of the hidden layer, respectively. In the neural network, the output of the hidden layer is taken as the input of the output layer. Assuming that the dimension of the output vector corresponding to each sample is *y*, the final output representation is shown in formulae (4) and (5):

(4) $$\begin{array}{c} \hat{y}=\text{softmax}\left(HW_{hy}+b_{y}\right), \end{array}$$

(5) $$\begin{array}{c} \text{softmax}\left(x_{m}\right)=\frac{e^{x_{m}}}{\sum_{k}e^{x}k}. \end{array}$$

### 3.2. Transformer Neural Network Translation Model

Attention mechanism is used for machine translation tasks. Encoder or decoder layers are directly used for attention, which reduces the transmission path of information. In addition, this attention approach can directly mine the semantic combination relationship between words inside sentences, and treat it as a semantic whole, making better use of word combination and even phrase information in translation, and better encoding semantic matching target language words. The final experimental results show that with the reduction of computation and the improvement of parallel efficiency, the translation result is also improved. Transformer is the encoder and decoder, respectively. The encoder maps the natural language sequence into a hidden layer, that is, the mathematical expression containing the natural language sequence. The decoder is responsible for remapping the hidden layer to a natural language sequence. First of all, text is typed in Transformer for embedding. That is word embedding processing. Text information is transformed into high-dimensional real vector. In order to identify the sequential relationship between statements, position embedding is introduced, and linear transformation of sine and cosine functions is used to provide position information for the model.

The article "Short Sequence Chinese-English Machine Translation Based on Generative Adversarial Networks of Emotion" was published in 2022. Journal: Comput Intell Neurosci.

In the encoder of Transformer, *N* = 6, that is, there are six layers, and each layer includes two sublayers, as shown in Figure 2. The first sublayer refers to the multihead self-attention mechanism, which is mainly used to calculate the self-attention value. The second sublayer is a simple fully connected network. Residual networks are added to each sublayer, and the output of each sublayer is shown in the equation (6):

(6) $$\begin{array}{c} \text{LayerNorm}\left(x+\text{Sublayer}\left(x\right)\right), \end{array}$$

where Sublayer(*x*) represents the mapping of input *x* by the sublayer. To ensure dimension consistency, all sublayers and word embedding layers have the same output dimension. Transformer decoder is also composed of *N* = 6 layers, each layer includes three sublayers. The first sublayer is masked multihead self-attention, which is also used to calculate self-attention. However, because it is a generation process, there is no result at time *i* greater than *i*, and only at time less than *i*, so mask processing is required. The second layer is the encoder input, related to attention calculation. The third sublayer is also a fully connected network, the same as encoder's sublayer fully connected network. The encoders and decoders of the Transformer model do not contain cyclic neural networks or convolutional neural networks, so it is impossible to capture sequence information. For example, if *K*, *V* are scrambled in line, the result will be the same after attention. However, the sequence information is very important, representing the global structure of the sequence, so the relative or absolute position information of each word of the sequence must be used.

### 3.3. Generative Adversarial Network

The core idea of generative adversarial network is derived from the Nash equilibrium of game theory, which is a two-player game in which the sum of the interests of both sides is a constant. The generation problem is regarded as the competition and game between generator and discriminator networks: the generator generates synthetic data from a given noise (generally evenly distributed or normally distributed), and the discriminator distinguishes the generator's output from the real data [42]. The former tries to produce more realistic data, while the latter, in turn, tries to better distinguish real data from generated data. Thus, the two networks make progress in the confrontation and continue to fight after progress. Then the data obtained from the generative network is more and more perfect, approaching the real data, so that the desired data can be generated. The antagonistic network judges that the text belongs to positive or negative emotion, and the final output results include that the emotional state that is more consistent with the language characteristics. The overall architecture of the model is shown in Figure 3.

The article "Short Sequence Chinese-English Machine Translation Based on Generative Adversarial Networks of Emotion" was published in 2022. Journal: Comput Intell Neurosci.

The left half of Figure 3 is made up of generator *G* and discriminator *D*. Among them, *G* is our neural machine translation model, which generates target sentences. *D* discriminates between the sentences generated by *G* and the artificial translation sentences, and generates feedback results. The right part carries out strategy gradient training for *G*, and the final feedback is provided by *D* and *Q*,, where *Q* is BLEU value. The model of generator *G* is similar to the model of neural machine translation. Generator *G* defines the method of generating the target sentence y, given the source statement *x*. The generator uses exactly the same architecture as the neural machine translation model. It is noteworthy that we do not assume a specific model structure for generator *G*. In order to verify the effectiveness of the proposed method, the generator adopts Bi-LSTM and Transformer. Since the length of the target sentence generated by the generator is not fixed, the discriminator model CNN fills the generated sentence to a certain extent and converts the target sentence into a sequence with fixed length *T*, which is the maximum length of the output target sentence of the generator. Given the source sentence sequence [*x*_1_, *x*_2_, ..., *x*_*T*_] and the target sentence sequence [y_1_, *y*_2_, ..., *y*_*T*_], the source matrices for the source sequence and the target sequence are, respectively, established as shown in the following expressions:

(7) $$\begin{array}{c} X_{1:T}=x_{1};x_{2};...;x_{T},\left(x_{t}\in R^{k}\right),\\ Y_{1:T}=y_{1};y_{2};...;y_{T},\left(y_{t}\in R^{k}\right). \end{array}$$

When *l* words undergo convolution operation, a series of feature graphs are generated, as shown in the formula (8):

(8) $$\begin{array}{c} c_{ji}=\sigma \left(BN\left(w_{j}⊗x_{i:i+l-1}+b\right)\right), \end{array}$$

where ⊗ represents the sum of principal element multiplications, *b* is the offset term, and *σ* is the activation function. Apply the BLEU value to the generator as a specific target. For the target sequence *y*_*g*_ generated by the generator and the real target sequence *y*_*d*_, by calculating the n-element syntax accuracy of the generated target sequence *y*_*g*_, the calculated result *Q*(*y*_*g*_, *y*_*d*_) is used as the feedback of the final generation. In order to facilitate the fusion of *D* and *Q*, the value range of *Q*(*y*_*g*_, *y*_*d*_) is 0–1, the same as the output of the discriminator. The objective of generator *G* is defined as maximizing the expected feedback from the beginning state of the generated sequence, and the objective function is shown in the formula.

(9) $$\begin{array}{c} J\left(\theta \right)=\sum_{Y_{1:T}}G_{\theta }\left(Y_{1:T}|X\right)\cdot R_{D,Q}^{G_{\theta }}\left(Y_{1:T-1},X,Y_{T},Y^{*}\right), \end{array}$$

where *θ* is the parameter in generator *G*, *Y*_1:*T*_=*Y*_1_, *Y*_2_, ..., *Y*_*T*_ is the target sequence generated by generator, *x* is the source sentence sequence, *Y*^*∗*^ is the real existing target sentence sequence. The action value function from the source sentence sequence *X* given by *R*_*D*,*Q*_^*G*_*θ*_^ to the target sequence indicates that the generated feedback is accumulated from the state. The action value function is calculated by combining the actual probability estimation output of discriminator *D* with the output of BLEU objective function *Q* as feedback.

The article "Short Sequence Chinese-English Machine Translation Based on Generative Adversarial Networks of Emotion" was published in 2022. Journal: Comput Intell Neurosci.

## 4. Experimental Analyses

The experimental models were done on the Tensor Flow framework and then run on the GPU. When the model ran ten evaluation tests on the test set and the model performance did not improve, we stopped training the model. BLEU value is used as the evaluation index of translation results. In order to ensure the fairness of the experiment, 1 million sentence pairs are randomly selected from the LDC corpus as training data, and the source and target statements are encoded by byte pair encoding, respectively. About 36,000 words are generated in the source language and 32,000 words in the target language. Select NIST04 as the test set and NIST02 as the verification set. The hidden neural units of both the encoder and decoder are set to 512, and the dimension size of word embedding is also set to 512 dimensions.

For the Transformer translation model, the basic structure of the model is used without any changes. We set the dimension size for word embedding to 512 dimensions, Dropout to 0.1, and multiple to 8. Both encoders and decoders have a six-layer network structure. For Bi-LSTM translation model, the number of hidden units of encoder and decoder is set to 512, and the dimension size of word embedding is also set to 512 dimensions. Dropout is not used to train the Bi-LSTM translation model.

### 4.1. Baseline Experimental

It can be clearly seen from Figure 4(a) that the BLEU score of RNN model is low, indicating that the translation effect generated by the original RNN is not very good. This is because in the original RNN translation model structure, the Encoder needs to compress the whole source language sentence into a fixed dimension vector, and then the Encoder-Decoder decodes the whole target language sentence from it. This requires that the fixed dimensional vector contain all the information of the source language sentence, which is obviously difficult to achieve, so it becomes the performance bottleneck of the original RNN as a machine translation model. Although Bi-LSTM and Transformer models are better than traditional RNN models, the effect is still not ideal.

The article "Short Sequence Chinese-English Machine Translation Based on Generative Adversarial Networks of Emotion" was published in 2022. Journal: Comput Intell Neurosci.

Bi-LSTM model, due to the internal bidirectional time extraction of features, has a stronger timeliness of features, so it reaches the highest 35.74 in NIST04, and the average BLEU value is 34.06. Transformer, due to its own attention mechanism, well explores the potential connection between different time points, and the features obtained have stronger internal connection, and the overall effect is significantly improved. In order to clearly show the changes of the three groups of experiments, we used another way to express the experimental results, as shown in Figure 4(b).

### 4.2. Generative Adversarial Network Model Experiment

According to the basic experiment, we select Bi-LSTM and Transformer, two models with better performance, to join the generative adversarial network. Experimental results were grouped according to the size of training parameters *λ* of generating adversarial network (0, 0.7, 0.8, 1.0). As can be seen from the experimental results in Figure 5, when the parameter *λ* of generating adversarial network is 0.7, the Bi-LSTM model achieves the best effect and the highest average value is 35.88. According to the changes of four curves, the experimental model in this paper conforms to objective laws.

Transformer is the most outstanding model in all fields of artificial intelligence at present, and has been greatly improved after the introduction of GAN. As can be seen from Figure 6, the lowest BLEU introduced by Transformer model into generative adversarial network is 41.4, higher than the average of other models. When the parameter *λ* value of generated admission-network is 0.8, the model achieves the best result of 43.14 and the average value of 42.73. From the overall experimental results, BLEU values of Bi-LSTM and Transformer models have basically the same change rule with parameter *λ*, both of which are nonlinear changes. It is important for our subsequent improvement. As an expression mode closely related to culture, language deserves more features and models.

The article "Short Sequence Chinese-English Machine Translation Based on Generative Adversarial Networks of Emotion" was published in 2022. Journal: Comput Intell Neurosci.

## 5. Conclusion

With the development of economic globalization, communication between countries, industries, and people of all countries are becoming more frequent and closer. Language is the tool of communication between people. How to quickly and accurately realize the free conversion between different languages is vital. Machine translation is an important research direction in natural language processing, and the development of deep learning related technologies has improved the methods and performance of machine translation. Machine translation as an efficient tool for language conversion, is of great practical significance in translating different languages into equivalent languages while preserving original semantics. Aiming at common neural machine translation models, this paper combines generative adversarial network with machine translation and improves the translation effect of translation models through adversarial training of generative adversarial network. In this paper, classic neural network model and attention-based Transformer model are studied. Then, Bi-LSTM model and Transformer model are added with generative adversarial network, respectively. Through the addition of generative adversarial network, the newly constructed model is analyzed and studied. Through the adversarial idea of generative adversarial network, certain feedback is obtained from discriminator *D* and acted on generator *G* to improve the translation effect of the translation model, get two emotional attributes of opposite polarity, and the effectiveness of the improved analysis method is verified through the final experiment. There are many hidden forms of emotion in language, and it is difficult to find the deep meaning of language by ordinary models, which is also the biggest advantage of the model in this paper.

## Figures and Tables

**Figure 1:** Expansion diagram of RNN internal structure.

**Figure 2:** Transformer encoder structure diagram.

**Figure 3:** Generate an adversarial network diagram.

**Figure 4:** BLEU value diagram of baseline experiment. (a) Baseline model BLEU histogram. (b) Baseline experimental grouping diagram.

**Figure 5:** Experimental results of Bi-LSTM + GAN.

**Figure 6:** Experimental results of transformer + GAN.

## Data Availability

The raw data supporting the conclusions of this article will be made available by the authors, without undue reservation.
